This article has been retracted.

# Pure Uterine Lipoma: A Report of a Rare Entity

**DOI:** 10.7759/cureus.20444

**Published:** 2021-12-15

**Authors:** Kayan S Alfarra, Ayesha A Aldhamer, Hiba S Aldubaib, Majd A Majoun, Aisha S Alrammah, Fedaa S Alshehri, Hanan M Mughallis, Awatif J Almalki, Ghadeer G Basakran, Areej M Alayed, Ghadah A Fallatah, Shahad F Alanazi, Amnah S Alamri, Omnia O Abuzahirah, Faisal Al-Hawaj

**Affiliations:** 1 College of Medicine, Batterjee Medical College, Jeddah, SAU; 2 College of Medicine, Princess Nourah Bint Abdul Rahman University, Riyadh, SAU; 3 College of Medicine, Dar Al Uloom University, Riyadh, SAU; 4 College of Medicine, Ibn Sina National College for Medical Studies, Jeddah, SAU; 5 College of Medicine, King Abdulaziz University, Jeddah, SAU; 6 College of Medicine, Umm Al-Qura University, Mecca, SAU; 7 College of Medicine, King Saud Bin Abdulaziz University for Health Sciences, Riyadh, SAU; 8 College of Medicine, Medical University of Lublin, Lublin, POL; 9 College of Medicine, Northern Border University, Arar, SAU; 10 College of Medicine, Imam Abdulrahman Bin Faisal University, Dammam, SAU

**Keywords:** case report, postmenopause, computed tomography, genital tract bleeding, uterine lipoma

## Abstract

Abnormal genital tract bleeding is a commonly encountered complaint in general practice. It has a wide range of etiologies and the spectrum depends on the reproductive status of the patient. While it represents a small proportion of genital tract bleeding, endometrial carcinoma is the main concern in postmenopausal women with abnormal genital bleeding. However, the majority of cases are due to benign etiologies. We present the case of a 65-year-old woman who presented to the outpatient department complaining of vaginal bleeding and lower abdominal pain for the last two months. The patient did not report any use of hormonal replacement therapy. Her last Pap smear was five years ago and it yielded no abnormal cells. On examination, the patient appeared obese with a body mass index of 35 kg/m^2^. Abdominal examination revealed a palpable pelvic mass that was firm and non-tender. The patient underwent an abdominal computed tomography scan which demonstrated a well-defined oval-shaped homogeneous fat attenuation mass lesion within the uterine wall with no evidence of invasion. Such findings were suggestive of uterine lipoma. The patient underwent a total hysterectomy and bilateral salpingo-oophorectomy. Histopathological examination of the specimen confirmed the diagnosis of pure lipoma. After six months of close follow-up, the patient had no active complaints. Pure uterine lipoma is an exceedingly rare benign neoplasm of the uterus. It may present with an abdominal mass and abnormal genital bleeding. Awareness of the clinical and radiological features of this tumor is crucial to avoid unnecessary surgeries in asymptomatic patients.

## Introduction

Abnormal genital tract bleeding is a common presenting complaint in family medicine and gynecology clinics. The etiology of genital tract bleeding depends largely on the patient’s age and reproductive status [1]. Postmenopausal bleeding occurs in up to 10% of women and accounts for 5% of gynecology visits [2, 3]. Despite that the genital tract bleeding is a worrisome complaint in postmenopausal women as it is the primary sign of endometrial cancer, the majority of patients have benign conditions like endometrial atrophy [1]. Prior research showed that the causes of postmenopausal genital tract bleeding, in descending order, included endometrial polyp, atrophy, fibroids, and endometrial carcinoma [4]. Here, we present the case of a postmenopausal woman who presented with abnormal genital tract bleeding that was diagnosed as having a pure uterine lipoma, a rare clinical entity.

## Case presentation

We present the case of a 65-year-old woman who presented to the outpatient department complaining of vaginal bleeding for the last two months. She reported that the bleeding was small in amount and did not occur daily. The bleeding was associated with lower abdominal pain. The bleeding was not related to the sexual intercourse. She did not report any changes in her urinary or bowel habits. There was no history of anorexia, weight loss, or fever.

The patient reached menopause at the age of 53 years. Her last Pap smear was five years ago and it yielded no abnormal cells. The patient did not report any use of hormonal replacement therapy. She was sexually active with her husband. The patient had three spontaneous vaginal deliveries with the last being 35 years ago. The past medical history was remarkable for asthma and glucose-6-phosphate dehydrogenase deficiency. She had no history of surgical procedures. She was a retired school teacher. She never smoked or consumed alcohol. Her family history was unremarkable.

On examination, the patient appeared obese with a body mass index of 35 kg/m^2^. The vital signs were within the normal limits. Abdominal examination revealed a palpable pelvic mass that was firm and non-tender. The speculum examination showed a normal vagina and cervix. Digital rectal examination was normal. The hormonal analysis revealed a normal level of prolactin (10 ng/mL), thyroid-stimulating hormone (2.5 mU/L), and normal thyroid hormones levels. Further, a basic laboratory investigation revealed anemia with a hemoglobin level of 10.2 g/dL (Table 1).

**Table 1:** Summary of the results of laboratory findings

Laboratory Investigation	Unit	Result	Reference Range
Hemoglobin	g/dL	10.2	13.0–18.0
White Blood Cell	1000/mL	7.2	4.0–11.0
Platelet	1000/mL	390	140–450
Erythrocyte Sedimentation Rate	mm/hr.	12	0–20
C-Reactive Protein	mg/dL	5.2	0.3–10.0
Total Bilirubin	mg/dL	0.8	0.2–1.2
Albumin	g/dL	3.9	3.4–5.0
Alkaline Phosphatase	U/L	51	46–116
Gamma-glutamyltransferase	U/L	16	15–85
Alanine Transferase	U/L	20	14–63
Aspartate Transferase	U/L	19	15–37
Blood Urea Nitrogen	mg/dL	10	7–18
Creatinine	mg/dL	0.9	0.7–1.3
Sodium	mEq/L	137	136–145
Potassium	mEq/L	3.8	3.5–5.1
Chloride	mEq/L	102	98–107

The patient underwent an abdominal computed tomography scan for better evaluation of the palpable lower abdominal mass. The scan demonstrated a well-defined oval-shaped homogeneous fat attenuation mass lesion within the uterine wall with no evidence of invasion. Such findings were suggestive of uterine lipoma (Figure 1).

**Figure 1:** Axial (A) and coronal (B) CT images of the pelvis demonstrate a well-defined fat-density lesion (arrow) in the uterus. CT: Computed tomography

The findings were discussed in the multidisciplinary oncology meeting. The decision for a total abdominal hysterectomy was planned. The patient agreed on having the surgery. Subsequently, the patient was prepared for a laparotomy operation. During exploration, the uterus was enlarged and the ovaries were atrophic. Total hysterectomy and bilateral salpingo-oophorectomy were performed. No complications occurred during the surgery. The skin incision was closed and the patient had an uneventful recovery. Histopathological examination of the uterus confirmed the diagnosis of pure uterine lipoma (Figure 2).

**Figure 2:** Microscopic histopathological image of the resected tumor demonstrates mature adipose cells in keeping with pure lipoma.

Postoperatively, the patient had complete resolution of the abdominal pain. She was discharged on the fourth postoperative day. After six months of close follow-up, the patient had no active complaints.

## Discussion

We present the case of a postmenopausal woman with pure uterine lipoma that manifested as abnormal genital tract bleeding. Uterine lipoma is one of the lipomatous groups of tumors of the uterus that include pure lipoma, lipofibroma, angiomyolipoma, liposarcoma, and others. Such a group of tumors is uncommon with an incidence of less than 1 per 1,000 women [5]. However, a pure uterine lipoma is exceedingly rare with few reported cases in the medical literature.

Several hypotheses have been suggested to provide an explanation for the development of uterine lipomatous tumors. The most widely accepted hypothesis proposes that such tumors arise as a result of metaplasia of the smooth muscles into adipose tissue [6]. However, other hypotheses include fatty degeneration of uterine smooth muscles or abnormal differentiation of the uterine mesenchymal cells [7].

The typical location of uterine lipoma is the corpus, as in the current case. However, the uterine lipoma may arise in the subserosal or submucosal location. Ultrasound examination and computed tomography scan may provide a clue to the diagnosis [8]. Magnetic resonance imaging has a higher accuracy as it can distinguish lipoma from other similar lesions like a liposarcoma. In the present case, we did not require such imaging because the patient was planned for surgical resection of the uterus given her symptoms [7].

As in the present case, uterine lipoma usually develops in postmenopausal women aged between 50 and 70 years [5]. The majority of uterine lipomas are asymptomatic and found incidentally. However, our patient had a history of genital tract bleeding and abdominal mass that were concerning for a malignancy. The prognosis of pure uterine lipoma is excellent as the risk of malignant transformation is negligible [8]. Surgical intervention may not be needed in asymptomatic patients and close observation is sufficient [5].

## Conclusions

Pure uterine lipoma is an exceedingly rare benign neoplasm of the uterus. It may present with an abdominal mass and abnormal genital bleeding. Awareness of the clinical and radiological features of this tumor is crucial to avoid unnecessary surgeries in asymptomatic patients. However, surgical resection may be required in symptomatic patients with an excellent prognosis.
